The article "Integrated Methods for Household Greywater Treatment: Modified Biofiltration and Phytoremediation" was published in 2023. Journal: J Environ Public Health.

# Integrated Methods for Household Greywater Treatment: Modified Biofiltration and Phytoremediation

**DOI:** 10.1155/2023/7778240

**Published:** 2023-01-28

**Authors:** Tolossa Waqkene, Seid Tiku Mereta, Amare Terfe, Wuhib Zeine Ousman

**Affiliations:** ^1^Department of Public Health, Dawo District Health Office, Southwest Shoa, Woliso, Ethiopia; ^2^Department of Environmental Health Science and Technology, Institute of Health, Jimma University, P.O. Box 378, Jimma, Ethiopia; ^3^Department of Environmental Health Science, College of Medicine and Health Sciences, Arba Minch University, P.O. Box 21, Arba Minch, Ethiopia

## Abstract

Most countries around the world have experienced water scarcity in recent decades as fresh water consumption has increased. However, untreated wastewater is routinely discharged into the environment, particularly in developing countries, where it causes widespread environmental and public health problems. The majority of wastewater treatment method publications are heavily focused on high-income country applications and, in most cases, cannot be transferred to low and middle-income countries. An experimental study was conducted to evaluate the performance efficiency of pilot-scale physicochemical and biological treatment methods for the treatment of household greywater in Jimma, Ethiopia. During the experiment, grab samples of greywater were taken from the combined treatment system's influent and effluent every 7 days for 5 weeks and analyzed within 24–48 hours. Temperature, DO, EC, turbidity, TDS, and pH were measured on-site, while BOD, COD, TSS, TP, TN PO_4_^−3^-P, NO_3_-N, NH_4_-N, Cl^−^, and FC were determined in the laboratory. During the five-week pilot-scale combined treatment system monitoring period, the combined experimental and control system's mean percentage reduction efficiencies were as follows: turbidity (97.2%, 92%), TSS (99.2%, 97.2%), BOD_5_ (94%, 57.4%), COD (91.6%, 54.7%), chloride (61%, 35%), TN (68.24, 42.7%), TP (71.6%, 38.7%), and FC (90%, 71.1%), respectively. Similarly, the combined experimental and control systems reduced PO_4_^−3^-P (12.5 ± 3 mg/L), NO_3_-N (4.5 ± 3 mg/L), and NH_4_-N (10.19 ± 2.6 mg/L) to PO_4_^−3^-P (3.5 ± 2.6 mg/L, 7.5 ± 1.6 mg/L), NO_3_-N (0.8 ± 0.5, 3.6 ± 2.3 mg/L), and NH_4_-N (7 ± 2.9 mg/L, 15.9 ± 3.9 mg/L), respectively. From the biofiltration and horizontal subsurface flow constructed wetland combined systems, the experimental combined technology emerged as the best performing greywater treatment system, exhibiting remarkably higher pollutant removal efficiencies. In conclusion, the combined biofiltration and horizontal subsurface flow constructed wetland treatment system can be the technology of choice in low-income countries, particularly those with tropical climates.

## 1. Introduction

Increasing population growth and industrialization have led to an exponential rise in global water pollution in recent decades [1]. It is expected that by 2050, the world population will have risen to approximately 9 billion people [2]. Both developed and developing nations experience this global population growth, though the latter is more significant. In turn, this leads to a rise in fresh water demand and a decline in fresh water resources due to population growth and improvements in people's daily life. Due to this, there is a rise in the amount of wastewater produced, a need for more sanitation methods, and an overall rise in environmental and public health issues [2, 3].

Thus, currently, two-thirds of the world's population lives in water-stressed areas for at least one month out of the year and by 2025, half of the world's population will be living in water-stressed areas, increasing the demand for direct and indirect wastewater reuse for survival [2, 4]. As a result, water scarcity, poor water quality, and water-related disasters in general have emerged as the most pressing global issues pertaining to current and future water resources [2, 3].

Used water from a household, municipality, or industry that contains 99% water and 1% suspended and dissolved solids is referred to as wastewater [2]. Household wastewater is wastewater produced at the household level by human activity [5], which is categorised into greywater and blackwater [6]. Greywater is the wastewater produced in bathtubs, showers, hand basins, kitchen sinks, dishwashers, and laundry machines which accounts for the majority of the flow (50–80%) [2, 7, 8].

In developing countries, particularly in urban and periurban areas, greywater is frequently discharged untreated into street drains or onto open ground, primarily ending up in rivers, resulting in oxygen depletion, eutrophication, and microbial and chemical contamination of soil and aquatic systems [2, 9, 10]. In the absence of treatment, this greywater contributes an excessive and frequently unwanted amount of chemicals and pathogenic microorganisms, endangering the environment, food safety, and human health [11–13]. Each year, at least 1.8 million children under the age of five die due to water-related diseases, accounting for roughly 17% of all deaths in this age group [2]. This suggests that the situation in developing countries is getting worse [2, 14]. Hence, these pollutants should be removed before greywater is reused or released into the environment in order to protect the environment and public health.

Over the last two decades, numerous studies have been conducted to assess the energy, economic, and environmental benefits of recycling greywater through nature-based solutions (NBSs) such as constructed wetlands (CWs) and biofiltration (BF) [15–19]. These technological advancements imitate how greywater is treated in nature. Therefore, one clever way to reclaim and lessen the detrimental effects of untreated greywater on the environment and public health is to encourage nature-based greywater treatment solutions.

For nearly two centuries, biofiltration, which was inspired by nature's self-purification of water, has been used for community water treatment [15]. It is a well-known natural water treatment method that uses various types of filter media beds to remove various pollutants from greywater [15, 20–22]. Studies have shown that different types of pollutants can be removed from greywater using filter media made of sand, charcoal, avocado peels, corn cobs, and gravel [15, 21–29]. This could happen through straining, sedimentation, ion exchange, adsorption on media surfaces, and microorganisms that degrade pollutants [30, 31].

Constructed wetland is the other recently proved and efficient greywater treatment technology that employs macrophytes such as vetiver grass [1, 32]. In comparison to conventional treatment systems, constructed wetland is a nature-based greywater treatment system that has been effective, affordable, and environmentally sound for repurposing greywater [17, 32]. The vetiver system, which is based on vetiver grass (*Chrysopogon zizanioides* L. Roberty), has been successfully used as a phytoremediation tool to remediate greywater due to its demonstrated extraordinary and unique morphological and physiological characteristics [1, 33]. When compared to other plants, vetiver plant was a candidate for removing a variety of pollutants, particularly N and P from greywater [1, 10, 17, 34]. The interaction of vetiver, microorganisms, and substrates results in natural processes (biological, chemical, and physical) that can remove pollutants from greywater [30].

Thus, the purpose of this study was to evaluate the treatment efficiency of physicochemical and biological methods for removing pollutants from household greywater by combining biofiltration with a constructed wetland planted with vetiver grass and to justify the potential efficiency of such technology as an alternative treatment method in the climatic conditions of Ethiopia.

## 2. Materials and Methods

### 2.1. Study Area

The study was conducted in a single purposefully chosen household in Jimma town, Southwest Ethiopia (Figure 1). Jimma town, the capital of the Jimma Zone, is located in Oromia Regional Administration, Southwest Ethiopia, at a latitude of 7°40′49″°N and a longitude of 36°49′18″°E; it is 354 kilometers from Addis Ababa and has an elevation of 1718 m. The study area receives a mean annual rainfall of 1529 mm, which is caused by a long and short rainy season. The town's average monthly temperature ranges from 11.7°C to 27.6°C [35].

### 2.2. Study Design and Period

Experimental study design was conducted in Jimma University at Laboratory of Environmental Health Sciences and Technology from June to July 2021.

### 2.3. Experimental Set Up and Operating Conditions of the Greywater Treatment System

The combined pilot-scale modified biofiltration and horizontal subsurface flow constructed wetland system was installed in a single purposefully chosen household with seven inhabitants (Figure 2). The specific area was located at a longitude of 036°50′48.129″°E and a latitude of 07°40′58.759″°N, with an altitude of 1734 m ASL. The variables considered for the combined system's design and construction were the required water quality, hydraulic loading rate (HLR), hydraulic retention time (HRT), substrate, and vegetation [36, 37].

#### 2.3.1. Layout and Configuration of the Pilot-Scale Treatment System

Figures 2 and 3 depict the layout, configuration, and other characteristics of the combined biofiltration and constructed wetland system, which are summarized in Table 1. A 200 L polyethylene filtration tank with an area of 1.8 m^2^ (*r* = 0.23 m, *h* = 1 m) was installed as secondary treatment and filled with different layers of filter media [10]. The sand and gravel filter media used in the filtration system were obtained from a quarry or gravel pit. The other filter materials were collected from the environment because they are easily accessible. Before filling the tank, the collected materials were thoroughly washed with tap water and dried in the sun. 

At the bottom of the barrel, a cast iron pipe with 8 mm diameter holes spaced 20 mm apart was inserted. Then, the bottom 20 cm layer was filled with drainage gravel aggregates of size 10 cm. The second layer, 10 cm thick, was filled with 5 cm corn cob, which is an important biosorbent for removing toxic organic and inorganic pollutants from water. The third layer was 10 cm thick avocado peel, with a size of 4 cm. Charcoal 3 cm in size was layered in the fourth layer, which was about 10 cm thick. The top most layer of about 20 cm was 0.8-1 cm grain size sand. The storage capacity above the sand was set to 30 cm in order to provide the required head to produce the design flow through the bed shown in figure 2 [38–40].

The flow rate of water through the filtration system was determined to estimate the capacity or amount of water that the filter could produce in liters per hour or liters per day. The flow rate was determined using a 1 L measuring cylinder and a stopwatch (discharge rate). Based on the following equation, the average time taken by the water through the filter bed to fill a 1 liter measuring cylinder for three replications was determined [41].

(1) $$\begin{array}{c} Flow\;rate\left(Q\right)=\frac{V}{t}\text{,} \end{array}$$

where *Q* = flow rate, *V* = volume of the effluent, and *t* = discharge time through the filter media.

Based on previous literature, a surface area of 0.65 m^2^ (Figure 3) was determined for the pilot-scale constructed wetland [42, 43]. It was constructed from a board measuring 1.3 m in length, 0.5 m in width, and 0.40 m in depth and was aligned to 1% slope to maintain the hydraulic gradient [9, 43–46]. The interior of the wetland was lined with high-density polyethylene (0.1 mm) plastic sheet [46]. As a substrate, it was layered with sand and gravel [44]. The bottom 20 cm was filled with 2-3 cm gravel aggregates. A 10 cm thick layer of 0.8–1 cm sand was filled in the middle, and the topmost 10 cm was filled with fine sand (0.1–0.4 mm). To avoid creating insect breeding sites, the water surface was kept 5 cm below the upper part of the substrate. In order to achieve a uniformly distributed flow, 10 cm gravel was placed in the inlet and outlet zones of each cell [44, 46–48].

#### 2.3.2. Installation of Inlet and Outlet Pipes

Polypropylene random (PPR) pipe with 3/4 inch diameter and 0.75 m length was installed to the inlet and outlet of each system to transport greywater from the treatment system's collection tank to the filtration and CW system (Figure 3). The greywater was then gravity-fed from the feeding tank to the filtration and wetland system. The pipeline at the inlet of each biofiltration and wetland system was fitted with a gate valve to control the flow of greywater and to prevent raw greywater from entering each CW during the hydraulic retention time (HRT). As a result, the amount of greywater entering the biofiltration cell was adjusted using a stopwatch and a graduated glass container; i.e., the HLR at the biofiltration's inlet was set to 0.4 m^3^/day [37].

At the CW inlet point, a 30 cm long PPR pipe with 7 mm diameter holes drilled every 5 cm was inserted. It was designed to ensure equal greywater flow distribution at the inlet of the horizontal CW, so that effluents from the filtration system run slowly through the porous fill media beneath the bed's surface in a more or less horizontal path until they reach the outlet zone. As an outlet pipe, a 1/2 inch PPR faucet was inserted 10 cm from the bottom of the CW. All of the pipes, valves, and the wetland system in general were checked twice a day to ensure proper greywater flow and system operation.

#### 2.3.3. Experimental Plant Selection and Establishment

In order to remediate greywater, the vetiver system, which is based on vetiver grass (*Chrysopogon zizanioides* L. Roberty), has been successfully used as a phytoremediation tool. This is because vetiver grass has been shown to have extraordinary and unique morphological and physiological characteristics when compared to other plants. It is the most effective species among the top three, including *Phragmites australis* and *Cyperus alternifolius.* Vetiver can withstand a wide pH range of 3.5 to 11.5, as well as extreme heat and cold (−14°C to 55°C) and salinity. Additionally, it was capable of absorbing significant amounts of potassium, phosphorus, and nitrogen. It has a high level of disease and pest resistance. Since it is sterile, it has no chance of growing into an aquatic weed [1, 33]. Along with these qualities, this plant was chosen due to its high biomass, root density and depth, ease of propagation, capacity to absorb or transform pollutants, tolerance of eutrophic conditions, ease of harvesting, and potential for using harvested material [1, 42].

We obtained 240 green, young vetiver grass samples from the Jimma University College of Agriculture and Veterinary Medicine nursery. Each grass had at least 2-3 well-developed leaves and roots. Five vetiver tillers were then planted in the substrate of the horizontal subsurface flow system (HSSFCW) with their roots and leaves pruned to 20 cm and 30 cm, respectively. The second CW was left vegetated-free as a control to measure the effectiveness of the planted CW [46, 49, 50]. The planting took place in April. The wetland beds were filled with tap water immediately after the plantation was completed, and watering of the wetland with rain water and tap water continued for two months, until the wetland plants adapted to the environment and grew well [51]. Following that, after two months, the biofiltration and CW were supplied with 100 liters of greywater from the receiving tank on a regular basis to monitor the combined treatment system's performance efficiency [46]. Moreover, since it was a rainy season, covers were designed for HSSFCW to eliminate the effect of the rainfall throughout the experiment period.

### 2.4. Operation and Maintenance of the Combined Treatment System

#### 2.4.1. Operation and Maintenance of the Biofiltration System

Regular maintenance is required for a proper functioning of the greywater filters. Clogging is a frequent issue with biofiltration and can be caused by components of greywater, as well as any material that falls on the filter. In this case, the use of pretreatment is recommended. If clogging occurred, it could be remedied by carefully removing the cover layer(s) and mixing the filter media. Applying sand or gravel that has not been properly washed or that is of the wrong grain size may be the cause of persistent or frequent filter clogging. To ensure a good flow, the pipes should be regularly inspected [36, 51].

For organic filters, service life is an especially crucial factor to take into account. Because of the variety of filters and raw greywater material, there is no exact or specific rule for when filter media should be cleaned or refilled. However, greywater filtration by various types of filter media is checked and cleaned on average every 1–6 months and is maintained when significant head loss occurs, causing the filter to be out of service for 1-2 days [41, 52, 53]. UNEP/WECF [51] recommended that the sand and gravel media have to be replaced every 5–10 years.

#### 2.4.2. Operation and Maintenance of the Constructed Wetland System

Constructed wetland should be inspected on a regular basis to ensure their proper and ongoing operation. Pollutant removal in subsurface flow constructed wetland frequently relies on a diverse range of coexisting physical, chemical, and biological routes, which are critically dependent on numerous environmental and operational parameters [30, 31].

Experience has shown that early failure is likely to happen on many sites without the implementation of a maintenance regime. The problems that frequently occur include blockages of inlets and outlets, flow-regulating devices, siltation of storage areas, algal growth, and plant dieback. Depending on the pollutant loading, maintenance is expected to include cleaning or removal of sections of contaminated substrate and associated vegetation. If the vegetation has been destroyed, plant replacement may be required [42].

Once the plants are established, quick visual inspections are considered an important part of routine maintenance. The primary goals of these inspections are to maintain the desired plant communities within the wetland and to identify any problems before they become major problems. In addition to this, weeds and any patches of permanently dead plants should be removed, and bare patches should be replanted with transplants from healthy areas of the wetland [54].

There is debate over whether it is appropriate to harvest plants from artificial wetlands. The study conducted by Ellis et al. [42] indicates that there is no enough information available to decide whether or not harvesting is preferable [42]. However, Paul Truong [55] recommended harvesting of plants planted for phytoremediation two or three times a year for biomass utilization purposes or to export nutrients. Plant harvesting can improve removal efficiencies in treatment wetlands [56]. On the other hand, plant harvesting may also create an adverse impact on the biomass population attached to the plant roots, thereby decreasing the performance of constructed wetlands [57, 58]. Therefore, a general answer cannot be given, but plants need to be harvested for biomass utilization purposes or if they interfere with the operation or the maintenance activities of the treatment system [10, 58, 59].

#### 2.4.3. Productivity, Utilization Options, and Economic Potential of Vetiver Grass

Vetiver is a highly productive plant species. The dried, partially dried, or even fresh material that is obtained from the vetiver plant's harvested leaves, stems, and roots can be processed completely or in part. Vetiver's unprocessed products are used for animal feed (for dairy cows, cattle, sheep, horses, or rabbits), compost, thatching, agricultural use (as mulch), and biofuel. The plant's semiprocessed by-products are used as a raw material for furniture, pressed-fiber pots, ethanol production, botanical pesticides, hats, mats, and other handicrafts. The fully processed products are used for industrial products as well as fiberboard, herbal medicine, and essential oils [1, 10, 55, 60, 62].

### 2.5. Collection of Greywater

Greywater for this study was collected from a nearby kitchen, laundry, shower, and hand basin, primarily early in the morning when cleaning in most households was at its peak. The residents of the household were asked to manually dispose of greywater into the receiving tank through a 1 mm mesh sieve as primary treatment to prevent vegetable peels and food residue, plastics, papers, and hair from entering the treatment system [63]. Then, equal volumes of 25 L of real greywater from the kitchen, laundry, and shower/hand basin were collected and mixed in the feeding tank. The mixed 100 L greywater was then allowed to pass through a 3/4 inch PPR drain pipe into a 200 L polyethylene barrel filled with filter media [9, 51] and finally to the two mini-constructed wetland (Figure 3). The filtration valve was opened, and either the CW with vegetation or the control constructed wetland was opened to allow water to flow into the basin. When the CW with vegetation system pipe network was open, the control constructed wetland pipe network was kept closed, and vice versa. Initially, clear water from the overhead tank was flowed into the basin for two days prior to beginning testing for the horizontal system with greywater to ensure the overall system's functionality and to wash out the organic contents/debris within the filter media.

### 2.6. Sample Collection and Analytical Methods

Water samples were taken by the grab sampling technique every week from the inlet and outlet of the compartments of the treatment setup to determine the water quality [64]. The following sampling points were chosen based on the treatment system's configuration: sampling point 1 (raw greywater), sampling point 2 (after biofiltration), sampling point 3 (after HSSFCW), and sampling point 4 (after HSSFCW, after control CW). A total of 20 samples were collected throughout the monitoring period after the hydraulic retention time of 3 days [65, 66].

Temperature, dissolved oxygen (DO), pH, electrical conductivity (EC), total dissolved solids (TDS), and turbidity were measured on the spot with an HI 98290 multiparameter meter and an HI 7629829/10 probe (Hanna Instruments, Woonsocket, RI, USA). For at least 40 seconds, the probe was gently stirred in a 5 L bucket of water. Total suspended solids (TSS), biological oxygen demand (BOD_5_), chemical oxygen demand (COD), nitrate nitrogen (NO_3_-N), ammonia nitrogen (NH_4_-N), total phosphorous (TP), orthophosphate, and chloride (Cl) concentrations were all determined at Jimma University Environmental Health and Science Technology Laboratory using American Public Health Association standard methods (APHA) for water and wastewater examination. Total nitrogen (TN), however, was determined at the Jimma Agricultural Research Center (Table 2). As a result, with a thoroughly cleaned high-density polyethylene bottle (HDPE), 1 L of water for physicochemical and 300 ml of water in a sterile glass bottle for bacteriological analysis were sampled from each sampling point. In the case of physicochemical samples, the bottles were filled until they overflowed and then stoppered. These samples were sealed and labeled before being placed in an ice-filled cooler box and transported cool and dark to the lab, where they were stored at 4°C [67].

For treatment system efficiency, the percentage removal efficiency (%) of the pilot-scale treatment system was calculated for each of the wastewater parameters based on the mass flow difference between the effluent and influent relative to the influent [68].

(2) $$\begin{array}{c} Removal\;efficiency\left(\%\right)=\frac{Ci-Ce}{Ci}x\;100\text{,} \end{array}$$

where Ci = concentration of waste material in influent and Ce = concentration of waste material in effluent.

### 2.7. Statistical Analysis

Data entry and analysis were conducted using SPSS version 20 software. Significant differences in influent and effluent concentrations were determined using one-way ANOVA (analysis of variance) at *p* < 0.05 with *α* = 0.05. Mean and standard deviation determinations, as well as the analysis of variance method, were used to determine statistically significant differences between the data. The hypothesis of normality was verified via the Shapiro–Wilk test. As the condition of normality was not met for at least one sampling point (1, 2, 3, or 4) per variable, we analyzed the data with the Kruskal–Wallis H test combined with a post hoc pairwise comparison. Tukey HDS was used as a post hoc test to identify differences between means.

### 2.8. Operational Definition

#### 2.8.1. Duplicates

They are multiple experimental runs with the same factor settings [67].

#### 2.8.2. Control

It refers to the treatment in greywater with constructed wetland that duplicates all the conditions of the experimental treatment but contains constructed wetland with no vetiver grasses [67].

#### 2.8.3. Modified Biofiltration

In this study, a filtration system comprised of charcoal, avocado peels, and corncob was used in addition to sand and gravel.

### 2.9. Data Quality Management

For each analytical experiment, a standard reference material was used for calibration and quality assurance. All of the chemicals and reagents used in the laboratory tests were of analytical grade and of standard approved make. To achieve the best possible results, standard solutions and necessary reagents were prepared on a regular basis. Reagent blanks and analytical duplicates for the wastewater samples were also included to evaluate the analytical reproducibility, accuracy, and precision. Laboratory instruments were calibrated in the same way, using freshly prepared standard solutions. All experimental development, calibrations, standard preparations, experimental methods, data generation, and activity documentation were carried out in accordance with the APHA standard guideline for wastewater analysis [67].

### 2.10. Ethical Consideration

Ethical clearance was obtained from the Institutional Review Board, Institute of Health. Moreover, informed verbal consent was also received from the household where pilot setup was set up.

## 3. Results and Discussion

During the monitoring period, the pilot-scale biofiltration treatment system was operated at HLR of 0.4 m^3^/day, resulting in a HRT of 0.5 day or 12 hours for a filter barrel volume of 0.17 m^3^ (*r* = 0.23 m, *h* = 1 m). Simultaneously, the biofiltration effluent rate was measured to be 0.2 L/min, resulting in 0.288 m^3^/day. Moreover, the performance of combined systems of biofiltration and constructed wetland planted with and without vetiver grass in terms of contaminant removal was evaluated, based on physicochemical and biological parameters between inflow and outflow. The combined treatment system efficiency was also evaluated over the course of 3 months of system operation in terms of the feasibility of reclaimed greywater for non-potable reuse (Table 3).

It was also discovered that the vetiver grass displayed some common stress symptoms during the acclimatization period, such as leaf tip drying. Plant growth in the constructed wetland system, on the other hand, increased significantly when the system was filled with greywater effluent from the biofiltration system and changed color from pale green to dark green. This is because the nutrient supply provided by the greywater effluent allowed the plant to grow taller and survive the experiment. The plant can also withstand harsh climatic conditions as well as a wide pH and salinity range [1].

### 3.1. Physical Parameters

As presented in Table 3 and Figure 4, the mean temperature values for influent and effluent recorded during the monitoring period were range-bound between 21°C and 23°C, which is the optimum temperature for bacterial activity in the treatment system [30, 48]. This finding is in agreement with the results reported by Haddis et al. [70] and Selemani and Njau [71]. On the other hand, the lowest mean temperature (21.87 ± 0.4°C) recorded at the HSSFCW effluent could be attributed to the long HRT in the HSSFCW as well as shading effect of the vetiver grass surrounding the wetland [72, 73]. This low temperature result at the planted CW effluent is consistent with the results reported by Ling et al. [74]. Despite the fact that there was little difference in mean temperature across the treatment systems, the ANOVA test revealed that there was no significant difference in mean temperature (*p* > 0.05) across the combined treatment system categories. This trend might be attributed to the atmospheric weather conditions at the experimental site. Furthermore, the mean temperature score at the outlet of the HSSFCW treatment system was within the maximum allowable limit for effluent discharge into the environment. As a result, this could be regarded as a promising treatment option for environmental protection.

Turbidity in water denotes the presence of organic, inorganic, and suspended matter which affects water transparency [75]. According to our findings (Figure 5), mean water turbidity in raw GW of 951.6 ± 66.3 NTU was reduced to 26.7 ± 4.9 NTU in the combined biofiltration and HSSFCW system (*p*=0.001). The removal of this water turbidity was attributed to filtration and sedimentation, which were facilitated by the filter media in the biofiltration and the macrophytes roots, which reduce interspaces between gravel by forming dense filter media capable of removing suspended particles in the CW [30]. This may also be explained by the biofiltration treatment system's filter media depth [76]. The wetland was not fully utilized in removing these contaminants from the wastewater because the majority of the organic, suspended, and colloidal matter was filtered and left in the biofiltration.

In this study, high mean turbidity value (951.6 ± 66.3 NTU) was recorded during the monitoring period when compared to the results (444 NTU) reported by Oteng-Peprah and Nanne [77]. The difference in the findings might be due to the raw GW, which has the majority of its sources coming from the kitchen and laundry, as more turbid greywater is expected from these sources [77]. This finding is in agreement with the results reported by Edwin et al. [78]. The finding also supports the conclusion that the source, lifestyle, and daily activities of the household have a significant impact on the characteristics of greywater [79, 80]. Based on the findings obtained, the turbidity concentration at the HSSFCW's outlet was within the US Environmental Protection Agency's permissible domestic wastewater discharge limit.

The total suspended solids (TSS) in the influent and effluent of each compartment of the combined treatment system were used to calculate the amount of accumulated solids expected to be on the substrate as well as on the root of the vegetation for each compartment of the combined treatment system [81]. The TSS value (1073.5 ± 386.19 mg/L) recorded in the raw GW was found higher when compared to the results (537 mg/L) reported in [77]. The washing of clothes, shoes, vegetables, fruits, tubers, and a variety of other items that may contain sand, clay, or other materials could explain the difference in results [77]. Biofiltration and HSSFCW combination, on the other hand, resulted in TSS effluent of 10 mg/L over 3-day HRT, which is a value accepted by the US EPA standard for non-potable reuse of reclaimed domestic greywater. Analysis of variance revealed that, similar to water turbidity, the compartments of the treatment methods achieved a significant reduction in TSS (*p*=0.002).

Moreover, TSS removal was very efficient and consistent within the biofilter (96%), as shown in Tables 3 and 4, demonstrating the importance of the biofiltration as a secondary filter for TSS removal. The combination of the biofiltration with HSSFCW system in reducing TSS by 99.2% has proven to be very effective compared to the results of TSS (49%) reported in [82]. This value is also greater than that reported by Rahmadyanti et al. [83] who reported TSS removal of 90% in HRT of 3 days. This efficient removal of TSS from raw GW is critical for preventing clogging of the bed media in the HSSFCW system. Similar observation of mean TSS reduction was also reported by Ling and Apun [84] who studied biofilters combined with HSSFCW in the treatment of household greywater using ornamental plants in Kuching City, Malaysia. The greater performance of HSSFCW over control CW in TSS removal (Figure 5) could be attributed to the dense network of plant roots, particle sedimentation, and biodegradation of suspended particulates [30, 75, 85].

### 3.2. Chemical Parameters

Variation of pH in different parts of the treatment methods is presented in Table 3 and Figure 6. According to Oteng-Peprah and Nanne [77], pH is heavily influenced by the constituents of greywater and is typically in the range of 5–9. In this study, the raw GW had an acidic pH (4.86 ± 0.2), when compared to the results (6.05 ± 0.26) reported by Pakanati Chandra Sekhar Reddy and Arun [86]. The difference in results could be attributed to microorganisms decomposing the organic fraction of greywater. This acidic pH might have also resulted from greywater generated from the kitchen [87]. Bakare et al. [87] stated that kitchen GW had the lowest pH values when compared to other GW sources, which might be attributed to the rapid degradation of food particles and oils under anaerobic conditions.

In the HSSFCW, however, there was a slight increase in mean pH of 6.68 ± 0.4 (Figure 6). Similar observation of increase in mean pH was also reported by Ling and Apun [84] who studied biofilters combined with HSSFCW in the treatment of household wastewater using ornamental plants in Malaysia. This increasing trend of pH across the treatment system might be attributed to denitrification processes producing alkalinity [31]. As the mean concentration of DO was depleted (Table 3), the pH rose because denitrification took over and produced alkalinity. This pattern could also be attributed to the anaerobic decomposition of organic matter and the dissolution of bed granules in water [75]. Despite the fact that the mean pH score in the raw GW was 4.86 ± 0.2, the mean pH score at the HSSFCW outlet meets the US Environmental Protection Agency domestic wastewater discharge limit (*p* < 0.05).

Another important environmental parameter considered in this study was DO, which is important in wastewater treatment because it facilitates the degradation of organic matter by microorganisms [30]. As illustrated in Table 3 and Figure 4, the mean DO concentration in raw GW was low, since the raw GW had high organic content. However, the mean DO concentration increased slightly after passing of the raw GW through the biofiltration, to 0.47 ± 0.2 mg/L, and rose continuously as it passed through the HSSFCW to 0.51 ± 0.2, where it gained more oxidizing potential, whereas, in the control CW, the mean DO concentration was lower than that of the HSSFCW (0.42 ± 0.1). These findings are in agreement with those of Amiri and Tarik Hartani [67] who reported mean DO value of 0.26 mg in raw GW and 0.27 ± 0.86 mg/L in biofiltration and HSSFCW combined system.

Moreover, because DO was consumed for the degradation of organic matter in the biofiltration, the removal of these organic matter in the biofiltration resulted in less demand for DO in the CW, and thus an increase in DO was observed (Figure 4). Similar observation of a slight increase in DO mean concentration was also reported by Amiri and Tarik Hartani [66] who studied biofilter combined with HSSFCW in the treatment of household wastewater using ornamental plants in Malaysia. The observed decrease in mean DO from the outlet of the biofiltration (0.47 ± 0.1) to the outlet of the control CW system (0.42 ± 0.1) could be attributed to anaerobic microbial degradation of organic matter in the control CW [30, 66]. The increase in mean DO concentration after passing through the planted CW (0.51 ± 0.2), on the other hand, could be attributed to oxygen supply from vegetation roots [30, 88]. Moreover, intermittent feeding of the wastewater into the bed of the treatment system might have resulted in the reaeration of the system [89]. Despite the fact that slight differences in mean DO concentration were noted among the compartments of the combined methods, the mean DO difference between these treatment methods was not statistically significant (*p* > 0.05).

Total dissolved solids describe all solids (including mineral salts) dissolved in water. As illustrated in Figure 7, a slight increasing trend of TDS was observed from the influent of biofiltration (655.2 ± 33.4 mg/L) through the HSSFCW (904 ± 1.1.9 mg/L) and control CW (863 ± 62.67 mg/L) systems. This increasing trend of TDS through the combined treatment system could be attributed in part to the mineralization of organics or ion dissolution during the degradation of water pollutants in the compartments of the treatment system [30, 75, 78]. Significant mean difference (*p* < 0.05) of TDS between the compartments of the treatment system was also noted. The current study also revealed that the HSSFCW significantly reduced the mean chloride concentration of 170.55 ± 54.14 mg/L to 66.4 ± 11.21 mg/L, which could be attributed to filtration and sedimentation in the filter medium bed and HSSFCW's vegetation root network (*p*=0.004).

In this study, the mean concentration of EC value in the raw GW was 1259.2 ± 107.3 (Figure 7). This result is in agreement with the results reported in [90]. Furthermore, the mean concentration of EC value increased through the compartments of the combined treatment system from the biofiltration inlet to the HSSFCW and control CW outlets, with the HSSFCW having the highest mean EC value of 1601 ± 305.8 S/cm (Table 3). However, no significant difference in EC was observed (*p* > 0.05) across the compartments of the treatment method. The presence of high EC values throughout the field test indicates that the household greywater was possibly saline, which could be harmful to the environment if discharged untreated. This can be attributed in part to the mineralization of organic matter and dissolution of bed granules [30]. Despite an increasing trend in EC mean concentration across the combined treatment system, the values remained within the USEPA's allowable discharge limit.

Moreover, EC is a surrogate measure of TDS [91]. The type and nature of the dissolved cations and anions in the water influence the relationship between TDS and EC [92]. The average TDS/EC ratio for most wastewater ranges from 0.5 to 0.9 [93]. In this study, the TDS/EC ratio in the raw GW was determined to be 0.52, which is in agreement with the results reported in [94]. This relationship is not directly linear because the conductive mobility of ionic species varies depending on the nature of soluble ionic components, their concentration, and the temperature of water [95]. In general, the TDS : EC relationship is given by the following equation: TDS = *k* *∗* EC [91]. The value of *k* will increase along with the increase of ions in water.

The chemical parameters in greywater treatment systems are primarily made up of dissolved organic matter, which are expressed as BOD and COD. These variables are critical indicators of organic load in domestic greywater [95]. According to the findings of this study, the BOD_5_ and COD mean concentrations in the effluent of the combined biofiltration and HSSFCW were 71.3 ± 26.5 mg/L and 109.5 ± 57.9 mg/L, respectively, after 5 weeks of combined treatment system operation (Figure 8). Similarly, the combined biofiltration and HSSFCW's recorded mean percent reduction for BOD_5_ and COD was 94% and 91.6%, respectively, at a DO mean value of 0.51 ± 0.2 mg/L (Table 4). These values are lower than the results of BOD_5_ (99%) and COD (95%) at mean DO concentration of 3.4–4.6 mg/L reported by Ling et al. [74] who evaluated the performance of pilot-scale biofilters and constructed wetland with ornamental plants in greywater treatment. The difference in the findings could be explained by the filter medium used, organic matter content of the raw wastewater, and mean DO concentration available in the HSSFCW treatment system [96].

Furthermore, throughout the treatment system, mean COD concentration was found to be greater than mean BOD_5_ concentration (Figure 8). The presence of synthetic organic compounds found in domestic wastewater such as bleaches, surfactants, and beauty products, which can also be transformed into other by-products during the chemical and biological treatment of greywater, could explain the dominance of COD over BOD_5_ [96].

The average BOD_5_/COD ratio for most GW ranges from 0.31 to 0.71 [95, 97]. In this study, the BOD_5_/COD ratio in the raw GW was 0.9, indicating that more than 90% of organic matter in the wastewater could be biodegradable. This result is in agreement with the findings of Nyoman et al. [83]. In contrast to our findings, Albalawneh and Chang [95] reported BOD_5_/COD ratio of 0.58 which was much less than our findings. These disparities in results could be attributed to the characteristics and composition of the raw GW generated [96].

On the other hand, the COD : N : P ratio in raw GW in this study was found to be 100 : 1.1 : 1.6, indicating severe nitrogen deficiency in comparison to the optimal values of 100 : 20 : 1 as reported in [97]. As a result, the raw greywater used in this study had a balanced carbon and phosphorus composition in terms of what was required for bacterial growth, but with limited nitrogen. This finding is in agreement with the results reported in [78, 98]. In general, the combined biofiltration and HSSFCW effluent BOD_5_ and COD levels met the discharge standard and reuse limit for restricted irrigation.

Nitrogen transformation in HSSFCW and biofiltration is a multifaceted process that involves plant uptake, sediment adsorption, and microbial metabolism. According to Table 3, the mean concentration of TN in raw RG was 14.45 ± 13.3 mg/L, originating primarily from kitchen wastewater (Figure 9). This finding is consistent with that of Boyjoo et al. [90]. Moreover, the mean TN reduction in biofiltration, HSSFCW, and control CW effluent was 7.84 ± 2.8 mg/L, 4.59 ± 2.6 mg/L, and 8.28 ± 1.4 mg/L, respectively. In the biofiltration, the mean percent reduction of TN was 45.7%. This result was higher than the results (21.3%) reported by Amiri and Tarik Hartani [66] who evaluated combined biofilter and CW system for household wastewater treatment in Algeria's arid regions.

Similarly, the biofiltration + HSSFCW combined treatment system reduced TN by 68.24% at a mean DO concentration of 0.51 ± 0.2 mg/L and at a mean temperature of 21.7 ± 0.56°C (Table 4). This is lower than the result (87.6%) reported by Amiri and Tarik Hartani [66] who assessed an integrated biofilter + CW system for household wastewater treatment in Algeria's arid regions. The reason for this could be that nitrogen removal is frequently influenced by nitrogen species transformation, vegetation, media, wastewater type, and hydraulic retention times [99]. Despite the fact that differences in mean TN concentration were noted among the compartments of the combined methods, the mean TN difference between these treatment methods was not statistically significant (*p*=0.187).

During the monitoring period, NO_3_-N was found to increase from 4.5 ± 3.3 mg/L in raw GW to 5.3 ± 2.5 mg/L in the effluent of biofiltration, but it was found to decrease significantly in the effluent of HSSFCW (0.84 ± 0.5) (Figure 9). This pattern could be found in many studies on nitrogen transformation [100]. The increasing trend of NO_3_-N at the biofiltration filter outlet indicates that the nitrifying bacteria oxidized NH_4_-N to NO_3_-N [30]. On the other hand, according to Mtavangu et al. [75], nitrate removal in the HSSFCW is due to nitrification and denitrification, sedimentation and volatilization, and plant uptake; however, it is attributed to the denitrification and sedimentation process in the biofiltration medium column. Similar observation was also reported by Ling et al. [74] who studied biofilters combined with HSSFCW in the treatment of household wastewater using ornamental plants.

Moreover, the reduction of NH_4_-N in the combined treatment system was attributed to microbial metabolism, plant uptake, and its sorption to the sediment of the filter bed [30, 67]. Furthermore, unlike oxidized forms of N, ammonium nitrogen is removed from greywater via adsorption onto the wetland matrix's active cation exchange site [30].

Ye and Li [101] reported that DO concentration of ≥1.5 mg/L is essential for nitrification; however, denitrification occurs at ≤0.5 mg/L. Since the DO concentration in this study was 0.5 mg/L, denitrification was the dominant nitrogen removal process. As a result, it can be concluded that the main removal mechanism of organic nitrogen under anaerobic conditions (denitrification) in the treatment system was the reduction of NO_3_-N to molecular nitrogen (N_2_) [102]. On the other hand, Yin et al. [100] stated that, at pH < 8.5, denitrification of gaseous products was the main route of gas loss which was similar to the present study. The reason could also be attributed to the process of converting NH_4_-N to NO_2_-N, followed by the conversion of NO_2_-N to N_2_ gas via the denitrification process [31]. Furthermore, NH_4_-N could be removed through volatilization from wastewater when the pH of a system is >9. However, because the pH level in HSSFCW was 6.68 ± 0.36, volatilization of NH_4_-N might not have been the removal mechanism in this study [102].

As illustrated in Table 4, the mean concentration of TP in the raw GW was found to be 21.12 ± 2 mg/L, owing primarily to the washing detergents. This is consistent with the findings of Boyjoo et al. [90]. Furthermore, TP removal efficiency in biofiltration (39.1%) and HSSFCW (53.4%) was low when compared to the results reported by Amiri and Tarik Hartani [66] in the combined biofilter systems for the treatment of wastewater in Algeria. This low phosphorus removal in biofiltration and HSFCW could be attributed to the fact that the media used in these treatment systems (gravel, crushed stones, charcoal, avocado peels, and corn cob) do not typically contain large amounts of iron, aluminum, or calcium to facilitate phosphorus precipitation and sorption [103].

When compared to HSSFCW, phosphorus removal in the wetland with no vegetation was also low (Figure 10). As a result, the HSSCW removed the majority of the TP via sedimentation, vegetation uptake, precipitation, and filter material interception [30, 103]. Kadlec and Wallace [30] stated that orthophosphate is removed through bacteria and plant uptake, while precipitation and adsorption are responsible for the removal of all forms of phosphorus. Barker [104] also stated that the increased polyphosphate-accumulating organism (PAO) population in the wastewater treatment system as well as the excess phosphorus uptake within each PAO reduces the phosphorus content of the water.

Furthermore, the combined biofiltration and HSSFCW removed 71.6% of TP at mean temperature and pH value of 21.7 ± 0.6°C and 6.68 ± 0.36, respectively. This was less than the mean percent value of TP (87.72%) reported by Amiri and Tarik Hartani [66] in the household wastewater treatment by biofiltration combined with HSSFCW. The differences in the findings could be attributed to differences in the phosphorus concentration in the influent to the beds, as well as differences in the HRT, and material used to construct the beds [105].

### 3.3. Biological Parameters

In terms of FC, the mean FC counts in raw GW were significantly higher than expected (Figure 11). The raw GW had a mean FC count of 2.44 × 10^6^ CFU/100 ml, which was reduced by biofiltration to 1 × 10^6^ CFU/100 ml, and the HSSFCW further reduced FC count to 2.46 × 10^5^ CFU/100 ml. The presence of these bacteria in raw greywater could be caused by improper food handling in the kitchen, as well as direct contact with contaminated food, which has been identified as a source of enteric pathogenic bacteria [77, 106]. However, a significant reduction of FC (90%) was recorded at the outlet of the combined biofiltration and HSSFCW (*p*=0.001). This result is in agreement with the results of Ling et al. [74] and higher than the results reported by Nyoman et al. [82] who studied biofilters integrated with HSSFCW in the treatment of household wastewater.

The high removal of FC (90%) by the combined treatment system depicts the importance in safeguarding the public health from pathogenic microorganisms (Figure 11). According to Kadlec and Wallace [30], the mechanisms involved in the removal of FC are natural die-off, resource competition, sedimentation, predation, and photolysis. Because the compartments of the treatment systems were covered, photolysis was not the mechanism of removal of pathogenic microorganism in this study. However, adsorption and agglomeration in the biofilters could have resulted in significant filtration and sedimentation. Moreover, because many enteric bacteria cannot survive long outside of host organisms, the efficient removal of coliforms by the HSSFCW might also be attributed to the long duration HRT [107].

## 4. Conclusions

In Ethiopia, where the practice of discharging untreated greywater onto open ground or into water bodies is widespread, the application of efficient, affordable, less energy-intensive, and simple to operate greywater treatment methods is a major concern. In addition to being essential for environmental and public health protection, reusing treated greywater for non-domestic uses like irrigation, building projects, and ground water recharge can also open up additional opportunities.

The results of this study provide an overview of how well the combined treatment system performs in tropical regions like Ethiopia. It is anticipated to advance knowledge of how the combined treatment system with vetiver plants and fill media operated under the local climate in Jimma. The effect of pollutant loading on the treatment of domestic greywater is also important to consider. However, the treatment system's practical applicability is not as straightforward as claimed in various studies. Numerous issues could arise from failing to take into account even the most elementary technical tasks.

According to the raw greywater characterized in this study, the high pollutant load values, especially when compared to US EPA guidelines, were found to be an important indicator of the pollutant's potential impact on the environment and public health. However, the combined greywater treatment system showed an outstanding performance in remediating turbidity, TSS, chloride, BOD, COD, TP, TN, and FC. The effluent concentration of all greywater pollutants at the combined biofiltration and HSSFCW complies with the unrestricted discharge limit standard; however, BOD, COD, TDS, and FC comply with the restricted discharge limit standard set by US Environmental Protection Agency.

When the performance of the combined biofiltration and HSSFCW was compared to the performance of the combined biofiltration and control CW pilot-scale systems, the pollutant removal efficiencies of the combined biofiltration and HSSFCW system were found to be more efficient than the biofiltration and control CW combined system for all parameters during the monitoring period.

Because of the presence of aerobic and anaerobic phases, such a combination frequently optimized nitrogen and organics removal. Particularly, related to the biofiltration treatment system, the wider implementation of organic filter media might have shifted the existing research from external carbon addition to internal carbon supplies, thereby improving denitrification performances. For the greywater composition studied here, the process was run for any strength of greywater generated during the monitoring period, showing that the combined treatment system can be a load-tolerant greywater treatment technology, making it suitable for decentralized greywater treatment and greywater reuse in developing countries.

In general, it can be concluded that the treatment performance of the pilot-scale combined treatment system applied at Jimma town was very promising for the promotion and application of treatment system as an alternative greywater treatment system to protect the environment and public health. Ethiopia has favorable climatic conditions for the implementation of treatment system, and hence the technology can continue as competent solution to alleviate the inherent environmental problems associated with discharging of untreated greywater. Therefore, it is recommended to use the pilot-scale combined treatment system for wider application in different towns for the treatment of greywater in small communities/institutions such as universities, colleges, military camps, and farms.

The following suggestions and future research directions are provided based on the results obtained and the difficulties encountered during the experiment period:

- Managing household water pollution is a major concern for the government, policymakers, and the general public. Although there are a number of established and new methods for treating greywater pollution, ecologically based methods are largely preferred because of the broad acceptance among key stakeholders.
- Greywater must first undergo pretreatment before entering the combined treatment system at the plot level. Screening systems should be implemented to prevent the clogging of the treatment system by vegetable peels and other coarse materials, which are frequently found in many low-income communities that do not segregate waste and have primitive disposal methods.
- Principles for choosing vetiver plants and media were very effective. If pretreatment systems to lessen the strength of the greywater and a flow management system are in place, vetiver's performance in contaminant removal in a tropical climate can be trusted.
- Despite promising efforts thus far, there are still limitations in certain areas to demonstrate the efficacy of the pilot-scale combined treatment system in the treatment of emerging chemicals that defy conventional remediation methods in order to establish acceptable remediation strategies and ecological benchmarks for greywater treatment optimization.
- More research should be conducted on the microorganism profile, the mechanisms that could explain plant growth (plant biomass, role of nutrients, nutrient and heavy metal status in the roots and shoots of vetiver, and water use efficiency, among other things), and how toxic contaminants can be converted into less harmful substances to avoid pollution transfer from one source to another.
- It would be wise to conduct more research on the treatment system's long-term performance as well as the frequency of replacement and harvesting of vetiver plants.
- A brief three-month observation period was used for the study. It might not be all-inclusive. Therefore, more research should be done in different seasons while considering other factors, such as heavy metals and greenhouse gas (GHG) emission.
- Future research should also concentrate on examining different organic media, the proper ratio, and the filter life.
- Finally, it would be interesting to analyze the sustainability of the pilot-scale combined treatment system process and optimize it while taking the possibility of treatment system clogging into consideration.

## Figures and Tables

**Figure 1:** Map of Ginjo Guduru kebele showing the pilot-scale treatment system installation area.

**Figure 2:** Design of system flow diagram of the combined treatment system.

**Figure 3:** Installation of the process flow diagram of the pilot-scale combined treatment system.

**Figure 4:** Mean influent and effluent temperature and DO values among the treatment methods measured in the field for pilot-scale greywater treatment.

**Figure 5:** Mean influent and effluent turbidity and TSS values among the treatment methods measured in the field for pilot-scale greywater treatment.

**Figure 6:** Mean influent and effluent pH values among the treatment methods measured in the field for pilot-scale greywater treatment.

**Figure 7:** Mean influent and effluent EC and TDS values among the treatment methods measured in the field for pilot-scale greywater treatment.

**Figure 8:** Mean influent and effluent BOD_5_ and COD values among the treatment methods measured in the field for pilot-scale greywater treatment.

**Figure 9:** Mean influent and effluent total nitrogen, nitrate nitrogen, and ammonia nitrogen values among the treatment methods measured in the field for pilot-scale greywater treatment.

**Figure 10:** Mean influent and effluent TP and orthophosphate values among the treatment methods measured in the field for pilot-scale greywater treatment.

**Figure 11:** Mean percent reduction of fecal coliform counts in the influent and effluent of the treatment methods measured in the lab for pilot-scale greywater treatment.

**Table 1:** Summary of main characteristics of pilot-scale biofiltration and HSSFCW system.

Characteristics	Experimental biofiltration system	Experimental CW system
Flow pattern	Downward flow BF	HSSF
Configuration	Multilayer BF	One-stage CW
Substrates	Gravel, sand, corn cob, avocado peel, charcoal	Gravel and sand
Bed dimension	*r* = 0.23 m, *h* = 1 m	1.3 m × 0.5 m × 0.4 m
Bed depth	0.7 m	0.40 m
Surface area	1.8 m^2^	0.65 m^2^
Type of wastewater	Greywater	Effluent from BF
Design flow per day	0.4 m^3^	0.4 m^3^
Type of feeding/loading	Intermittent	Intermittent

**Table 2:** Summary of sample analysis methods.

Parameters	Analysis method	Setting	Reference
Turbidity	Nephloturbidimeter method 2130 B	On-site	[67]
Temperature	Multiparametric probe method 2510		
pH			
EC			
DO			
TDS			

TSS	Gravimetric method 2540C, 2540D	Lab	[67]
BOD_5_	Azide modification of Winkler method 5210 B		
COD	Open reflex, titrimetric method 5220 D		
Chloride	Argentometric method 4500 B		
TP	Stannous chloride method 4500 D		
PO_4_^−3^-P	Stannous chloride method 4500 D		
TN	Kjeldahl digestion method		
NO_3_^−^N	Phenoldisulphonic acid method		
NH_4_-N	Nesslerization method		
FC	MFM method 9221 B		

**Table 3:** Greywater characteristics (mean and standard deviation) (*n* = 5).

Parameters	Unit	Influent concentration/raw GW used as feed	Effluent concentration			[69] guideline for non-potable reuse of GW (unrestricted)^*∗∗*^
			Treated using biofiltration	Treated using CW with V. grass (BF + CW)	Treated using control (BF + control)	
pH	Numeric	4.86 ± 0.2	5.37 ± 0.6	6.68 ± 0.36	5.85 ± 0.45	6.5–8.4
Temperature	°C	22.75 ± 0.8	22.18 ± 1	21.72 ± 0.6	21.87 ± 0.4	—
DO	mg/l	0.27 ± 0.1	0.47 ± 0.2	0.51 ± 0.1	0.42 ± 0.1	Must be present
Chloride	mg/l	170.55 ± 54	143.23 ± 51.67	66.4 ± 11.21	110.69 ± 13.57	<70
EC	*μ*S/cm	1255.2 ± 107	1564 ± 166	1601.8 ± 306	1480.4 ± 345	<700 *μ*S/m
TDS	mg/l	655 ± 33	803.8 ± 62	904 ± 102	863 ± 63	<450
Turbidity	NTU	951.6 ± 66.3	139.74 ± 53.79	26.71 ± 4.9	76.12 ± 50.61	<30
TSS	mg/l	1073.5 ± 386.19	41.4 ± 29	8.76 ± 8	30 ± 21.7	<30
BOD_5_	mg/l	1184.4 ± 121.3	628.5 ± 83.6	71.34 ± 26.46	502.9 ± 35.5	<30
COD	mg/L	1297 ± 88.2	719.9 ± 68.5	109.5 ± 57.99	587.4 ± 79.6	<100
TP	mg/l	21.12 ± 2	12.87 ± 2.35	6 ± 1.15	12.94 ± 2	<10
PO_4_^−3^-P	mg/l	12.51 ± 3	11.19 ± 4	3.53 ± 2.6	7.5 ± 1.6	<10
TN	mg/L	14.45 ± 13.3	7.84 ± 2.8	4.59 ± 2.6	8.28 ± 1.4	<10
NO_3_^−^N	mg/l	4.52 ± 3	5.31 ± 2.5	0.84 ± 0.5	3.64 ± 2	<5
NH_4_-N	mg/l	10.19 ± 2.6	10.99 ± 4	7.05 ± 2.9	15.92 ± 3.9	—
FC	CFU/100 ml	2.44 × 10^6^ ± 1,777,245	1 × 10^6^ ± 314,038	2.46 × 10^5^ ± 83,570	6.98 × 10^5^ ± 348,784	<1000

Each value of the parameter is described as mean value ± SD. pH, potential of hydrogen; DO, dissolved oxygen; TN, total nitrogen; EC, electrical conductivity; TSS, total suspended solids; TDS, total dissolved solids; NH_4_-N, ammonium nitrogen; NO_3_^−^N, nitrate nitrogen; COD, chemical oxygen demand; BOD, biochemical oxygen demand; PO_4_^−3^-P, phosphate phosphorus; FC, fecal coliform; USEPA, United States Environmental Protection Agency; BF, biofiltration. ^*∗*^Because Ethiopia lacks a standard discharge limit for domestic wastewater, we used the USEPA's effluent discharge limit standard. ^*∗∗*^Unrestricted effluent discharge limit.

**Table 4:** Mean percentage reduction of the effluent concentrations or treatment performance (%) of the integrated biofiltration and HSSFCW systems (mean over total service time).

Parameters	Mean concentration out of each treatment unit					% removal			Total % removal	
	Unit	Influent and effluent				BF	CW	Control	BF + CW	BF + control
		Raw GW	BF	CW	Control					
Turbidity	NTU	951.6	139.7	26.7	76.1	85.3	80.9	45.5	97.2	92
TSS	mg/L	1073.5	41.4	8.8	30	96	78.7	27.5	99.2	97.2
BOD_5_	mg/L	1184.4	828.5	71.3	502.9	46.9	88.6	20	94	57.4
COD	mg/L	1297	719.9	109.5	587.4	44.5	84.8	18.4	91.6	54.7
Chloride	mg/L	170.6	143.2	66.4	110.7	16	53.6	22.7	61	35
TN	mg/L	14.45	7.84	4.59	8.28	45.7	41.45	5.3	68.24	42.7
TP	mg/L	21.12	12.87	6	12.94	39.1	53.4		71.6	38.7
FC	CFU/100 ml	2.4 × 10^6^	1 × 10^6^	3.26 × 10^5^	7.4 × 10^5^	58.1	68.1	58	89.9	71.4

Each value of the parameter is described as mean percentage reduction. TN, total nitrogen; TSS, total suspended solids; COD, chemical oxygen demand; BOD, biochemical oxygen demand; TP, total phosphorus; FC, fecal coliform; BF, biofiltration; CW, constructed wetland; HSSFCW, horizontal subsurface flow constructed wetland.

## Data Availability

The data used to support the findings of this study are available from the corresponding author upon request.
